This article has been retracted.

# A Comprehensive Review of Various Diabetic Prediction Models: A Literature Survey

**DOI:** 10.1155/2022/8100697

**Published:** 2022-04-12

**Authors:** Roshi Saxena, Sanjay Kumar Sharma, Manali Gupta, G. C. Sampada

**Affiliations:** ^1^CSE Department, Gautam Buddha University, Greater Noida, India; ^2^Cedargate Technologies, Kathmandu, Nepal

## Abstract

Diabetes is a chronic disease characterized by a high amount of glucose in the blood and can cause too many complications also in the body, such as internal organ failure, retinopathy, and neuropathy. According to the predictions made by WHO, the figure may reach approximately 642 million by 2040, which means one in a ten may suffer from diabetes due to unhealthy lifestyle and lack of exercise. Many authors in the past have researched extensively on diabetes prediction through machine learning algorithms. The idea that had motivated us to present a review of various diabetic prediction models is to address the diabetic prediction problem by identifying, critically evaluating, and integrating the findings of all relevant, high-quality individual studies. In this paper, we have analysed the work done by various authors for diabetes prediction methods. Our analysis on diabetic prediction models was to find out the methods so as to select the best quality researches and to synthesize the different researches. Analysis of diabetes data disease is quite challenging because most of the data in the medical field are nonlinear, nonnormal, correlation structured, and complex in nature. Machine learning-based algorithms have been ruled out in the field of healthcare and medical imaging. Diabetes mellitus prediction at an early stage requires a different approach from other approaches. Machine learning-based system risk stratification can be used to categorize the patients into diabetic and controls. We strongly recommend our study because it comprises articles from various sources that will help other researchers on various diabetic prediction models.

## 1. Introduction

Diabetes is a disease that is caused due to excessive amount of blood sugar in it. Our body needs energy, and glucose is one of the main sources of energy to build the muscles and tissues of the body. Generally, unhealthy lifestyle and lack of exercise are the main causes of type 2 diabetes in people. The presence of a large amount of sugar in the blood causes diabetes. Sometimes, the pancreas is unable to convert the food into insulin; thus, sugar remains unabsorbed, which causes diabetes. Diabetes can affect kidney, eyes, nervous system, blood vessels, and so on. Diabetes is of three types. First is juvenile diabetes [1], which occurs mostly in children and destroys the cells which produce insulin in the pancreas. Second is type 2 diabetes, which generally happens after the age of 40 because of lack of exercise and unhealthy lifestyle. Diabetes is a type of disease that cannot be reversed but can be controlled with the help of medications, regular walk and exercise, and a proper diet. Type 2 diabetes [2] is also known as insulin-independent diabetes since patients are not injected with insulin after a gap of regular intervals, but in the case of type 1 diabetes, insulin is injected at a regular interval of time to the patient, so this is also known as insulin-dependent diabetes. The third type of diabetes [3] is gestations, which occurs during pregnancy due to the change of hormones, and this generally disappears after the delivery. There is one more condition, that is, prediabetes, in which the intake levels of sugar are on the borderline, and this condition can be reversed with the help of regular exercise and healthy lifestyle. In this paper, we have tried to predict diabetes using machine learning. Machine learning is a branch of artificial intelligence in which the machine tries to predict the outcome based on certain data and previous outcomes. Machine learning is of two types. First is supervised learning, in which data act as a teacher and the model is built around the dataset. Second is unsupervised learning, in which data trains itself by finding certain patterns in the dataset and labeling them. In recent years, many authors have published and presented their work on diabetes prediction by using machine learning algorithms. In this paper, we have studied various diabetes prediction methods using machine learning and presented a comparative study of a few methods in our paper. The objectives of our study are as follows:

1. To enrich ourselves with the various diabetic prediction models.
2. To evaluate and discuss the existing models based on classification accuracy.
3. To discuss the various attributes required for the prediction of diabetes.
4. To identify the research gaps in the existing literature.
5. To present a comparative study of various diabetic prediction models.
6. To collect more and more information about the prediction of diabetes in the primitive stage.

The idea that had motivated us to review the various diabetic prediction model is to address the diabetic prediction problem by identifying, critically evaluating, and integrating the findings of all relevant, high-quality individual studies. To achieve our motivation for this review process, we have studied various articles on diabetic prediction models, and we have taken those articles in this review process that have satisfied the following criteria:

1. Article must have discussed various predictive methods and machine learning algorithms for the classification of diabetes data.
2. Article must have discussed various preprocessing techniques to filter the noisy data.
3. Authors have validated their model against a few performance parameters such as sensitivity, specificity, accuracy, true positive rate, and true negative rate.
4. Predictive models were compared with the other existing diabetic prediction models.

The organization of the remaining paper is as follows: Section 2 discusses the rigorous literature review conducted by us during our review process.  Section 3 discusses various diabetic prediction models by different authors, followed by Section 4, which comprises a comparative analysis of different methods based on different comparative parameters.  Section 5 discusses the existing challenges and issues in various diabetic prediction models, and then a conclusion is presented at the end, that is, Section 6.

## 2. Literature Review

Healthcare systems offer customized services in broad-ranging areas to assist patients in integrating themselves into their regular routines of life. Diabetes mellitus is amongst the most significant severe problems in the medical profession. Classification is amongst the most significant decision-making methods in today's practical circumstances. The primary goal is to categorize the data as diabetes or nondiabetic and increase the classification accuracy. Machine learning in the diagnosis of diabetes is mostly about understanding patterns from the diabetes dataset which would be given. Machine learning in recent times has always been the developing, dependable, and supportive technology in the medical sector. This study is focused on the identification of diabetes types of patients based on personal and clinical information utilizing machine learning classifiers. This section contains a summary of the works suggested by different researchers during the last decade. It is beneficial to identify the shortcomings of suggested works in the field of diabetic patients' treatment regimen machine learning classifiers. Diagnosis of diabetes is a growing area of study. Sun and Zhang [1] have discussed a few deep learning methods and classification methods such as artificial neural network, decision trees, random forest, and support vector machine. Qawqzeh et al. [4] have implemented a logistic regression classification technique for the classification of diabetes data. Training data includes 459 patients, and testing data includes 128 patients. Classification accuracy achieved by the authors was 92% using logistic regression. The major disadvantage of the model was that it was not compared with the other diabetic prediction models and hence could not be validated. Tafa et al. [5] divided the dataset into 50% training set and 50% testing set. The model was proposed using a combination of naïve Bayes and support vector machine algorithms for diabetes prediction. Dataset was collected from three different locations, and the proposed model was validated on this dataset. Eight attributes were present inside the dataset, and it consisted of 402 patients, amongst which 80 patients were type 2 diabetic. Ensemble of naïve Bayes and support vector machine has achieved the accuracy of 97.6%, which is far better than the algorithms when run alone on the dataset, that is, Naïve Bayes achieving an accuracy of 94.52 and support vector machine achieving 95.52%. The authors have not mentioned any preprocessing technique to filter out any unwanted values from the dataset. Karan et al. [6] demonstrated a new method for diabetes diagnosis by designing a dispersed end-to-end three-level unavoidable healthcare system architecture utilizing artificial neural network (ANN) computing. At the most basic level, sensors and wearable devices are used to monitor vital indicators on the human body. At level 2, client-side devices such as PDAs and PCs serve as an arbitrator and communicator between both the primary and final levels. The third level end includes powerful desktop servers that provide customers with social welfare administrations and database operations. Applications of an artificial neural network are applied to diagnose illnesses at both the next and subsequent levels. Artificial neural network computations make the client and server model dependent on them. This method advances calculations and systems communications on the user and server sides by depending on the concept of illnesses. Sisodia and Sisodia [7] have applied Naïve Bayes, decision trees, and support vector machine learning algorithms on the Pima Indians Diabetes Dataset, and the maximum accuracy to predict the diabetes was achieved by Naïve Bayes classifier. A tenfold cross-validation technique was used by Sisodia in which the dataset was divided into ten equal parts: 9 parts were used for training, and the remaining part was used for testing. Evaluation parameters on which the diabetes was predicted were accuracy, precision, recall, and area under the curve. A review of various machine learning algorithms was presented by Hussain and Naaz [8] in which random forest, Naïve Bayes, and neural network were compared for accuracy. For evaluating these machine learning algorithms, the Matthews correlation coefficient was used by the authors. Kumari et al. [9] have worked on the Pima Indians Diabetes Dataset, applied Naïve Bayes, random forest, and logistic regression, and compared these three approaches with ensemble approach and model outperforms with ensemble approach with an accuracy of 79%. Olaniyi and Adnan [10] made use of deep learning, that is, neural network, which is a multilayer network and is feed forward. The authors implemented the algorithm on the Pima Indians Diabetes Dataset, and the dataset was divided in a way that 500 values were used for training purposes and 268 values were used for testing purposes. Dataset was normalized to achieve numerical stability before any preprocessing operations could be performed. To achieve the dataset normalization, all the dataset values were made to lie between 0 and 1 by dividing each attribute by their corresponding amplitude. The authors achieved the prediction rate as 82% accurate. Gupta et al. [11] worked with support vector machines and Naïve Bayes algorithms to classify the diabetic dataset. K-fold cross-validation model was used by the authors for training and testing purposes, and after applying both classification algorithms, the support vector machine classifier was performing better than the Naïve Bayes algorithm. Kandhasamy and Balamurali [12] predicted diabetes on a dataset that was taken from the UCI repository and applied a few machine learning algorithms such as J48, random forest, k-nearest neighbours, and support vector machine. The authors applied the above-said classifier once without preprocessing the dataset and once after the data is preprocessed. Preprocessing techniques were not discussed, with the mention of the fact that the dataset had some noise and was removed. The authors have evaluated the prediction on the basis of specificity, sensitivity, and accuracy. When the data was not preprocessed, the decision tree gave the highest accuracy of 73.82%, and with the preprocessing of the dataset, random forest achieved the highest accuracy of 100%. Choubey et al. [13] applied two feature selection methods named principal component analysis and linear discriminant analysis to extract significant features from the Pima Indians Diabetes Dataset. A comparative analysis of the feature selection method was also presented in the article. Few machine learning algorithms, that is, radial basis kernel, k-nearest neighbour, and AdaBoost, were also applied to the dataset for classification purposes. Perveen et al. [14] used the dataset from the Canadian primary care sentinel surveillance network. The attributes present in the dataset are sex, body mass index, triglycerides, fasting blood sugar, diastolic blood pressure, and systolic blood pressure. Classifiers used by the authors are decision tree, bootstrap, and adaptive boosting. Gujral [15] presented a survey on primary stages of type 2 diabetes diagnosis using machine learning algorithms and the identification of recurrently occurring complications associated with diabetic retinopathy and diabetic neuropathy. Numerous machine learning methods have been investigated and studied, including synthetic neural networks, essential parts, choice trees, hereditary computations, and fuzzy logic. The majority of the concerned literature makes use of the Pima Indians Diabetes Dataset as its informative index. Prediction of diabetes in the early stages is important because it reduces the lethal effects caused due to diabetes. The Writing Survey of Diabetes assumptions illustrates that a solo strategy to identifying diabetes is not an exceptionally urbane method for detecting diabetes early. The best results are obtained by combining classifiers such as support vector machine, principal component analysis, and genetic algorithms, as well as artificial neural networks. Mamuda and Sathasivam [16] made use of scaled conjugate gradient, Levenberg–Marquardt and Bayesian regulation, which are supervised machine learning classifiers. Data were split into testing and training sets, and Levenberg–Marquardt has obtained the best performance. Malik et al. [2] worked on a local dataset taken from a hospital in Germany and applied decision trees, k-nearest neighbour, and random forest on this locally available dataset. The probabilistic neural network was used by Soltani and Jafarian [17] for the detection of diabetes. 90% of the Pima Indians Diabetes Dataset was used as a training dataset, and the rest of the 10% was used for testing. The accuracy achieved was 89.56% for the training and 81.49% for the testing set. Tigga and Garg [18] worked on the Pima Indians Diabetes Dataset. Important features extracted from the dataset are blood glucose levels, number of pregnancies, and body mass index. Logistic regression was used to predict the accuracy using RStudio, and the accuracy achieved was 75.32%. Yuvraj and SriPreethaa [19] applied Naïve Bayes, decision trees, and random forest on the Pima Indians Diabetes Dataset. Moreover, in addition to machine learning algorithms, the information gain feature selection method was used to extract the significant features, and eight features were used instead of thirteen features. 30% of the dataset was used for testing purposes, and the authors have shown that maximum accuracy of 94% is being achieved by a random forest classifier. Rashid et al. [20] developed diabetes mellitus support systems, which run automatically using classification algorithms, captivating into versions the aforementioned issues and also mirroring the abilities of health experts who have faith that there is a strong correlation between the side effects of certain chronic illnesses and the glucose rate. The ramifications of this study may extend beyond merely categorizing diabetes mellitus patients. In this way, the main obligations are as follows: it makes use of certain free variables. Negi and Jaiswal [21] created their own dataset, which contains 102538 values and 49 attributes. In this dataset, approximately 64419 were diabetic patients, and the rest were nondiabetic. Missing values were replaced by preprocessing technique, and nominal data were changed to numerical data. The wrapper feature selection method, along with the ranker method, was used to select the relevant features from the dataset. Ensemble of a few classifiers was used further to achieve an accuracy of 72%. Mercaldo et al. [22] applied Bayes net, Hoeffding tree, random forest, j48, JRip, and multilayer perceptron on the Pima Indians Diabetes Dataset. Two feature selection methods, namely, greedy stepwise and best first, were used to select the significant attributes to increase the performance of classifiers. Only four attributes amongst eight were used. Four attributes were age, body mass index, diabetes pedigree function, and plasma glucose concentration. Hoeffding tree algorithm has achieved a recall value of 76.2% and a precision of 75.7%. Swapna et al. [23] applied convolution neural network and convolution neural network long short-term memory networks on Electrocardiograms, a private dataset that consisted of 142000 samples and has achieved an accuracy of 90.9%. Neither preprocessing nor any feature selection technique was applied in this dataset. According to Valasapalli et al. [24], type 2 diabetes mellitus (DM) is a long-lasting disease whose incidence has been steadily increasing worldwide. In India, about 30 million individuals have diabetes, and many more are at risk. Thus, early detection is necessary to avoid diabetes and its associated complications. The rationale for utilizing various methods for hypothetical type 2 diabetes determination grounded on the indicative study is to extend the disease's detection period by assessing suggestive features and regular habits, thereby enabling the estimation of type 2 diabetes without the use of clinical tests through predictive analysis. Today, an enormous amount of clinical knowledge is available about infections, their symptoms, the causes of illness, and their consequences for health. Due to the accuracy of these algorithms, the danger of type 2 diabetes may be predicted, which is critical for the medical sector. Lekha and Suchetha [25] created their own dataset, which was based on breath signals and consisted of 25 patients, amongst which 11 were healthy, five were type 1 diabetic patients, and nine were type 2 diabetic patients. Leave one cross validation was used for validation purposes, and evaluation parameters were ROC curve, which was approximately 96%. Mohebbi et al. [26] used a conventional neural network and multilayer perceptron neural network to detect diabetes on a dataset that consisted of 9 patients. Dataset was based on continuous glucose monitoring signal dataset. Six patients were used for training and validation, while the rest three were used for testing. The conventional neural network achieved the highest accuracy of 77.5%. Zou et al. [27] applied two feature selection methods on the Pima Indians Diabetes Dataset and Luzhou dataset collected from a local Chinese hospital. Three machine learning classifiers, that is, random forest, decision tree J48, and neural network, were run on both datasets. Two feature selection methods, namely, principal component analysis and minimum redundancy maximum relevance, were employed to reduce the number of attributes. The maximum accuracy achieved was 77.21% with random forest and minimum redundancy maximum relevance method. Ashiquzzaman et al. [28] have applied a deep neural network on the Pima Indians Diabetes Dataset. The deep neural network is composed of radial basis function, multilayer perceptron, and general regression neural network. Dataset was left unfiltered intentionally as the filtration was done by the deep neural network itself. The authors achieved an accuracy of 88.41%. The recurrent neural network was applied by Ramesh et al. [29]. 80% of the dataset is used for training purposes, and the rest 20% is used for testing purposes. The authors predicted accuracy for both types of diabetes and achieved 78% for type 1 and 81% for type 2 diabetes. An unsupervised deep neural network was proposed by Miotto et al. [30] to predict diabetes. Dataset consists of approximately 704857 patients. Data of 5000 patients were used for validation purposes, 76217 for testing, and the rest for training purposes. The authors have not used any feature selection technique. The evaluation parameter was the area under the curve, and the authors achieved an AUC of 0.91. Three different deep learning technique was applied by Pham et al. [31]. Dataset was collected by the authors from a hospital, and it consisted of 12000 values. One-sixth of the dataset was used for validation, two-thirds of the dataset for training purposes, and one-sixth for testing. Dataset was preprocessed and was reduced to 7191 values. The authors achieved the maximum precision value of 59.6%. A two-class neural network was applied by Somnath et al. [32] on the Pima Indians Diabetes Dataset. Dataset was preprocessed by using the mean values, and significant features were selected using the correlation attribute feature selection technique. The authors achieved the maximum accuracy of 83.3%. Diwani and Sam [33] applied decision tree and Naïve Bayes on the Pima Indians Diabetes Dataset. Accuracy was evaluated using Weka, and diabetes was predicted using Naïve Bayes with an achieved accuracy of 76.3%. According to Dremin et al. [34], ageing and diabetes both result in protein glycation and malfunction of collagen-containing tissues. Collagen mechanical and practical alterations accompany the development of a variety of pathological abnormalities distressing the skin, plasma vessels, and nerves, resulting in a variety of problems, increased impairment hazards, and a danger to life. Indeed, there are presently no noninvasive techniques for assessing glycation and related metabolic processes in biotissues or for predicting potential skin consequences, such as ulcers, for endocrinologists and clinical diagnosis. We propose a problem-solving method skilled at assessing the skin problems of diabetes mellitus at an early phase in this paper by using new photonics-based technologies, novel machine learning solutions, and decisive physiological features. The feasibility studies, as well as real testing on affected ones with diabetes and those who are nonaffected volunteers, demonstrate unequivocally that the method is capable of discriminating between affected, that is, diabetic and nonaffected, that is, control groups. Additionally, the internally developed polarization-based hyperspectral imaging method, along with the usage of an artificial neural network, opens up innovative avenues for the research and detection of growth-related illnesses. To increase the accuracy of a diabetic prediction model, Dwivedi [35] applied an adaptive neurofuzzy inference system, and a feature selection method named principal component analysis was used. Kamrul Hasan et al. [36] compared independent component analysis, correlation attribute feature selection, and principal component analysis feature selection method and applied Naïve Bayes, gradient boost, decision trees, random forest, multilayer perceptron, and AdaBoost. An accuracy of 78.9% was achieved using an ensemble of AdaBoost and gradient boost classifiers. Maniruzzaman et al. [37] worked on a dataset taken from National Health and Nutrition Examination Survey. Features were selected using logistic regression methods, and the random forest classifier gave the optimum result. Ramesh et al. [38] proposed a framework for automating the process of prediction of diabetes and made use of health devices such as smartwatches or a smartphone. The machine learning classifier used by the authors to classify the dataset is a support vector machine. Steps followed for prediction of diabetes are scaling down the attributes and then selecting the most significant one, imputation of null values followed by data augmentation. Performance parameters achieved by the authors are 83.20% sensitivity, 87.20% of specificity, and 79% accuracy. Vitals monitored by the authors in this paper are the amount of oxygen in the blood, pulse rate, diastolic blood pressure, medication status, systolic blood pressure, number of calories consumed in a day, count of the steps, and which type of activity is performed by the user. For consolidation of authentic information, which has to be provided to different cloud services vendors and transmission of information redirected towards the server, a mobile application was developed and installed in the smart wearable device, which directly transmits the user vitals to different cloud vendor platforms. Vital information was extracted by the mobile application system. Two vendor cloud services named Google fit and iHealth were used by the authors to extract the vital information obtained from smart wearable devices. Vitals extracted from smart devices are then visualized by the server to predict diabetes in a preliminary stage. The dataset used by the authors is the Pima Indians Diabetes Dataset. Some of the values in the dataset are missing and are being imputed by the author. The method through which values are imputed by the authors is not discussed in the paper. Imputation is followed by the standardization of the range of dataset values, and then only significant features were used that contribute highly to the prediction purpose. Feature selection methods used are chi-square, extra trees, and LASSO. The most important feature extracted were glucose, insulin, body mass index, and age. The maximum accuracy achieved was 79% through support vector machines.

## 3. Methods for Diabetes Prediction

### 3.1. Kamrul Hasan's Method

In this approach, a four-phase prediction method is used to predict diabetes. In the starting phase, preprocessing is performed on the dataset, which consists of rejecting the outliers and filling missing values. Outliers are values which are deviated from the normal observations. And there were certain missing values in the dataset, which were replaced by mean values instead of median values because of their greater tendency towards the attribute distribution. Outliers are abnormal observations which are deviated from the values of the dataset. Outliers need to be rejected because of the insensitivity of the machine learning algorithm towards distribution and range of attributes. Outliers can be calculated as follows:

(1) $$\begin{array}{c} p\left(x\right)=\left\{x,\text{ if }q1-1.5*IQR\leq x\leq q3+1.5*IQR,\text{ reject otherwise}\right., \end{array}$$

where *P* (*x*) is the mathematical formulation of outlier rejection [10], *x* is the instances of the feature vector that lies in the *n*-dimensional space, and *q*1, *q*3, and IQR are the first quartile, third quartile, and interquartile range of the attributes. Once the outliers were rejected, the authors found all the missing values of the dataset, and those values were filled with the mean of the particular attribute.

(2) $$\begin{array}{c} q\left(x\right)=\text{mean }\left(x\right),\text{ if }x=\frac{\text{null}}{\text{missed}},\;x\text{ otherwise.} \end{array}$$

In equation (2), *q* (*x*) is the mathematical formulation of mean imputation, and *x* is the instance of the feature vector that lies in the *n*-dimensional space. Attributes were rescaled to achieve standard normal distribution to reduce the skewness of the distribution. The authors employed independent component analysis [15], principal component analysis, and correlation-based feature selection technique to select the significant features, predicted diabetes by taking all features together, six significant features and four important features, and compared the result of the three-feature selection technique with 4, 6, and 8 features. Fivefold cross validation is used by the authors in which the dataset is divided into five equal parts, whereas four parts are used for training purposes and one part is used for testing purposes. It will be repeated 5 times, and in this manner, every part will be used for training as well as testing. Several classification algorithms such as a k-nearest neighbour, random forest, AdaBoost, multilayer perceptron, decision trees, gradient boost, and naïve Bayes were applied to the Pima Indians Diabetes Dataset by the author. The main evaluation parameters were sensitivity, specificity, and area under the ROC (receiver operating characteristics) curve. Mostly, all the classifiers have given their best result when the correlation-based feature selection method is employed and the data is in processed form. Classifiers have performed well when the authors have made use of six features instead of four or eight features. Diastolic blood pressure and diabetes pedigree function were discarded by the author, and the rest six were used for classification. Certain parameters were tuned in to optimize the evaluation parameters. Parameters that were optimized for k-nearest neighbour [17] by the authors are number of neighbours, leaf size, and distance function. The authors used the Gini criteria and best splitter for the decision tree. The grid search technique is applied to select the number of hidden layers while using a multilayer perceptron. Once the number of hidden layers is selected, the selection of the number of neurons in each hidden layer is to be done. Activation function [21], dropped neurons percentage neurons, neuron initializer, learning rate, size of the batch, epoch, loss function, and multilayer perceptron optimizer, is selected. Extensive experiments were carried out by the authors by applying diverse groupings of preprocessing technique and different machine learning algorithms to maximize the AUC parameter. The algorithm that gave the best results is proposed as a baseline model for evaluation of the proposed ensemble classifier. To ensemble the AdaBoost and gradient boost machine learning algorithm, soft weighted voting is done where the AUC is selected as the weight of that model for voting because it is unbiased to the class distribution. The authors have achieved an AUC of 0.95 with the ensemble of AdaBoost and gradient boost, preprocessing techniques with correlated feature selection method.

In this method, the author's main focus was on increasing AUC [10] parameter instead of increasing the accuracy of the system. Preprocessing the dataset and feature selection was the core concern, and it has helped the authors increase sensitivity and specificity. The method is a little bit time-consuming because the authors have tried many combinations of classifiers with preprocessed datasets and then with four, six, and eight features.

### 3.2. Quan Zou's Method

Quan Zou worked simultaneously on two datasets. One dataset is the Pima Indians Diabetes Dataset, and another dataset is from a local Hospital in Luzhou, China, which contains 14 attributes and approximately 68994 patient's data. The authors employed a two-phase detection method where the dataset was trained and two feature selection methods, namely, principal component analysis, minimum redundancy, and maximum relevance. They used three classifiers, that is, decision tree J48, random forest, and neural network. Decision tree classifier and random forest were run on Weka 3.9.4 to evaluate the prediction result while neural network model was implemented using MATLAB [16]. A fivefold cross-validation technique was employed by the authors to train and test each value. The authors made use of all the features of both datasets to predict diabetes and showed that the random forest method is predicting the disease with higher accuracy for the Luzhou dataset than the other two classifiers, and for the Pima Indians Diabetes Dataset, all the classifiers are giving the approximately same accuracy. The authors assumed that random blood glucose, fasting blood glucose, and blood glucose tolerance are the good parameters for diabetes prediction, the Luzhou dataset contains fasting blood glucose, and PIDD contains blood glucose tolerance attributes, respectively. When only the single feature glucose has been used by both datasets, J48 has better accuracy for the Luzhou dataset, and the results are not good for PIDD. Now, the authors used the minimum redundancy maximum relevance feature selection method to select the significant features. For the Luzhou dataset, features selected are height, fasting blood glucose, high-density lipoproteins, low-density lipoproteins, and breath, and for PIDD significant features are age, 2-hour serum insulin, and glucose. Again, for Luzhou, J48 has better performance, but the results were better when all the features were selected instead of only these five features. For PIDD, the best result was given by the random forest machine learning algorithm. Next, the authors made use of principal component analysis to extract the features. To extract the important features using PCA, statistical software for social sciences was used to analyse the factors. After analysing the composition matrix [24] and eigenvalues, five new features were selected for the Luzhou dataset and three for PIDD for conducting the experiment. When the three of the classifiers were run on the Luzhou dataset, accuracy was much less than the above-said methods. PCA is considered inappropriate for the Luzhou dataset by the author. When PCA [15] was used on PIDD, accuracy was better than that when using only a single attribute. The following experiments were designed by the authors to see the importance of other features for Luzhou datasets:

1. All the features except blood glucose were used for the prediction of diabetes.
2. Three features, that is, low-density lipoproteins, high-density lipoproteins, and blood glucose, were deleted, and the rest eleven features were used in the prediction. For those eleven attributes, the random forest was giving the maximum accuracy.
3. From all the analyses conducted by the author, the authors have stated that principal component analysis is not much suited for prediction purposes.
4. In the end, the authors have said that the three classifiers were performing much better with all the features collectively taken for prediction instead of selecting only a few significant features either through minimum redundancy and maximum relevance or through principal component analysis.

The maximum accuracy achieved was 80.86% for the Luzhou dataset through the random forest with all the features taken into consideration.

### 3.3. Nishith Kumar's Method

In this paper, the authors have assumed the medical data to be inherently structured, nonnormal, and nonlinear and therefore made use of three kernel-based Gaussian process classification against naïve Bayes, linear discriminant analysis, and quadratic discriminant analysis. Three kernels are linear, polynomial, and radial basis kernel [26], and then a comparative analysis of three kernels in the GPC and then the GPC is compared against naïve Bayes, LDA, and QDA. Evaluation parameters taken by the authors are sensitivity, specificity, accuracy, positive predictive value, negative predictive value, and receiver operating characteristics. Analysis of three types of kernels for a Gaussian process model has been done using Laplace approximation. A generalization of the logistic function is Gaussian process classification, and the authors have used the activation function as logistic regression [39]. Since there is no noise in the Gaussian process, it can be combined with an activation function; in this case, the authors have used the activation function as logistic regression. But it is too difficult to calculate the likelihood function using a logistic function. For this, the Laplace approximation to solve the binary class problem of the Gaussian process [24] has been used by the author. For binary class problems, a sigmoid function is used in the study, which is defined in equation (3) and *t* is the variable for which function is being computed.

(3) $$\begin{array}{c} \text{sigmoid }\left(t\right)=\frac{1}{\left(1+\exp\left(-t\right)\right)}. \end{array}$$

Steps implemented in this article for the prediction of diabetes are as follows:

1. Three kernels, namely, linear, radial basis, and polynomial, are compared for Gaussian process-based classification process to classify the patients into diabetic and nondiabetic. Laplace approximation has been used to implement the Gaussian-based process classification method.
2. Naïve Bayes, linear discriminant analysis, and quadratic discriminant analysis have been applied to the Pima Indians Diabetes Dataset, and evaluation parameters were compared with a 3-kernel-based Gaussian-based model.
3. A 5-fold and 10-fold cross-validation model was applied to the dataset, and sensitivity, specificity, accuracy, positive predictive value, negative predictive value, and AUC were evaluated for four of the classifiers. After the results were evaluated, naïve Bayes has performed the least, and radial basis Gaussian-based process classification has outshined all the classifiers.
4. Accuracy achieved was 81.97% with 10-fold cross validation, radial basis kernel GPC, sensitivity of 91.79%, specificity of 63.33%, positive predictive value of 84.91%, and negative predictive value of 62.5%.

The advantage of this system is its ability to fit in linear and nonlinear functions by handling uncertainty in unknown functions also. Probabilistic prediction can also be made through this model, but the main disadvantage of this model is to select a kernel for the correct representation of medical data.

### 3.4. Maniruzzaman's Method

In this article, the authors adopted four machine learning algorithms, that is, random forest [20], AdaBoost [23], naïve Bayes [11], and decision tree [13] on NHANES (National Health and Nutrition examination survey) dataset. This dataset contains 9858 patient's data, amongst which 760 are diabetic and 9098 are nondiabetic. There were certain missing values in the dataset, which the authors dropped from the dataset as a cleaning process. After dropping the missing values, there were 6561 respondents, amongst which 5904 were nondiabetic and 657 were diabetic. The authors selected the important features from the dataset by making use of the logistic regression model, *P* value, and odds ratio [40]. The probability of response is calculated from logistic regression [28] by making use of one or more predictions. The relationship between predictor and response is being measured through a logistic regression model, and a logit function is estimated. The equation of a logit function is defined as follows:

(4) $$\begin{array}{c} log\text{ it }\left(P_{j}\right)=log_{e}=\overset{k}{\underset{i=0\;}{\sum }}\beta_{i}X_{i}, \end{array}$$

where *P*_*j*_ is the probability of a patient being diabetic, 1 − *P*_*j*_ is the probability of being a nondiabetic, *i* = 0, 1, 2,…, *k*, unknown regression coefficient, and *k* is the total number of predictors or attributes (in this case, 14).

Using these regression coefficients in (4), the authors have found the *P* value and odds ratio of each of the features. *P* value is calculated from *t*-test for continuous variables and chi-square [31] test for discrete variables. Data is analysed by the authors through Stata version 14.10. Only those features are selected from the dataset by the authors whose *P* value is less than 0.005. The next step implemented by the authors was the splitting of the dataset into training and validation set. A 10-fold cross-validation model [29] is used in which the dataset is divided into ten equal parts where the nine parts are used as a training set, and the remaining one is used as a validation or testing set. This entire process is repeated 20 times, and the classification accuracy is calculated at each step. Then, an average of all classification accuracy is taken by the author. After selecting the significant features from the dataset and following a cross-validation model, the authors have applied four classifiers to the dataset, that is, naïve Bayes, random forest, decision tree, and AdaBoost. Evaluation parameters taken by the authors are accuracy, positive predictive value [24], negative predictive value [27], and *f*-measure. After conducting a few experiments, the accuracy achieved for K2, K5, and K10 models was 92.54%, 92.33%, and 92.75, respectively. The authors concluded that the best accuracy was given by random forest along with the logistic regression feature selection method.

### 3.5. V. Jackins Method

In this article, the authors have worked on three datasets together, diabetes, cancer, and heart disease. A two-step method is used by the authors in which the data in the dataset undergoes a cleaning process, and then the machine learning classifiers are applied to the datasets. Data preprocessing [18] includes replacing the missing values of the dataset with the null values and then checking the correlation between the features of the dataset. Correlation [27] helps in determining important features from the dataset. If two features are highly correlated, then one of the attributes from the dataset can be skipped while the other can be used for prediction purposes. In the next step, data is split into training and testing. 70% of the dataset is used for training purposes by the author, and the remaining 30% is used for testing purposes. Then, the naïve Bayes and random forest classifier are applied to the filtered dataset, and the evaluation parameters are compared. For diabetes, the authors have made use of the Pima Indians Diabetes Dataset. Dataset is analysed through Anaconda 4.1. The authors have checked to see if any categorical data in the form of true or false is present. If present, true is replaced by 1 and false by 0. When the missing values are filled by null values, the authors made use of the correlation coefficient [41], which can effectively measure the amount of corelationship between two variables. When the two attributes of the dataset are highly correlated, one of the attributes can be neglected so as to avoid repetition. After the calculation of the correlation of different attributes of the dataset, the authors created a correlogram matrix [13]. In the matrix, the blue colour represents positive coefficients while the red colour represents negative coefficients. The correlation coefficient and intensity of the colours are highly proportional. The range of the correlation coefficient is from −1 to +1. Value of +1 correlation coefficient indicates perfect positive correlation coefficient, and −1 indicates perfect negative correlation coefficient. After the calculation of the correlation coefficient, a confusion matrix is created by the author. Evaluation parameters on which the diabetes is predicted are accuracy, precision, recall, and *f*1-score. The accuracy achieved by the authors for the naïve Bayes algorithm is 76.72 and 74.46 for training and testing data, respectively, while for the random forest, it is 98.88 and 74.03 for training and testing data. The method applied by the authors consists of applying preprocessing techniques [42] by replacing missing values with null values and deleting those attributes from the dataset, which are highly correlated to each other. Classification algorithm random forest and naïve Bayes [11] are applied to the preprocessed dataset, and efficiency is calculated on the basis of accuracy. The performance of the algorithm proposed by the authors is compared with density-based spatial clustering of applications with noise (DBSCAN) algorithm and *k*-means clustering algorithm to measure the effectiveness of the algorithm. After comparison, the authors found the proposed algorithm to be better than K-means and DBSCAN. The main disadvantage of the method proposed by Jackins is the processing time, as a large amount of the data is taken for training and testing purposes. The advantage of the method is that it helps in diagnosing the disease with more accuracy.

### 3.6. N Sneha's Method

In this article, the authors have applied five classification methods, that is, random forest, k-nearest neighbour, support vector machine, naïve Bayes, and decision tree on a dataset which is downloaded from UCI repository and contains 15 attributes and 2500 values, although they took only 768 values for testing purpose. The attributes of the dataset taken by the authors are age, gender, plasma glucose fasting, postprandial plasma glucose, pregnancy, blood glucose level, blood pressure, skin thickness, insulin, body mass index, pedigree function, serum creatinine, serum sodium, serum potassium, and HBA1C. After determining the sensitivity [19] of the problem and dataset, the authors have selected a few relevant attributes from the dataset. The steps implemented by the authors for diabetes prediction [43] are as follows:

(1) Attributes and their importance are being analysed for the given problem.
(2) Attributes are being assigned a sequence number from 0 to maximum, where the maximum is the total number of attributes and 0 is the first attribute.
(3) Authors have taken the main attribute, which is responsible for causing diabetes, as an input attribute.
(4) Correlation of other attributes with the main attribute has been determined by them, and a value of correlation is generated. Value of correlation is generated using
  (5) $$\begin{array}{c} \text{Co}‐\text{relation value }=\left[{\text{attributes}}_{\text{max}}-\overset{n}{\underset{i=0}{\sum }}\text{ attribute }\left(x_{i}\right)\right]. \end{array}$$
Once the correlation values are calculated for a particular attribute, every other attribute undergoes the same value generation process. Once the correlation value of all the attributes is calculated, a comparison amongst all the attributes is made. If the difference between the correlated values of the two attributes is large, the attribute is considered less significant. By using this correlation, the best attribute from the dataset is selected and arranged in a significant order.
(5) Once the authors have determined the best attributes, classification algorithms can be applied to the dataset to improve the accuracy.

They have run the classification algorithms using the rapid miner tool, and the evaluation parameters taken by them are sensitivity, specificity, accuracy, precision, and recall. Accuracy achieved before her proposed method for support vector machine, random forest, naïve Bayes, decision tree, and k-nearest neighbour [44] was 77.73%, 75.39%, 73.48%, 73.18%, and 63.04%, respectively. After the proposed method, the authors have taken 11 features out of 15 based on their correlation. Features excluded by the authors are pregnancy, postprandial plasma glucose, serum creatinine, and HBA1C. By using the proposed method, the authors have achieved the highest specificity of 98.2% and 98% through decision trees and random forest, respectively.

### 3.7. Saumendra Mohapatra's Method

In this article, the authors have made use of only one classification algorithm, that is, multilayer perceptron, to detect diabetes at an early stage. Multilayer perceptron uses backward propagation method for classification of diseases. The authors have done preprocessing of data as a first step in the classification process. Pima Indians Diabetes Dataset has been used for classification and testing purposes. Division of the dataset is done in a manner that 70% of the dataset is used for training purposes and 30% for testing. Multilayer perceptron [16] makes reorganizing patterns for the classification of inputs and prediction of the stated problem. Before the dataset has been trained by the author, some random weights are used, and neurons of the neural network learn from the training dataset. The authors have left the missing value as missing only, and they were not replaced by any mean or median. 550 rows were used for training, and 218 were used for testing purposes. The authors have trained the network using the training data from the Pima Indians Diabetes Dataset. Eight input layers and four hidden layers were fed to the training network. Then, the testing and validation of the model is followed after training. Multilayer perceptron [45] is applied to the testing dataset, and then the authors measure the accuracy of the machine learning algorithm. Accuracy is calculated in (6) using the following formula:

(6) $$\begin{array}{c} \text{Accuracy }=\frac{TP+TN}{N}*100, \end{array}$$

where TP denotes true positive, TN denotes true negative, and *N* denotes the total number of values in the dataset.

The authors have a classification accuracy of 77.5%. Experiments are performed using the RStudio tool. The main drawback of the method is that no preprocessing of the data has been done on the dataset. The authors have made use of missing values as well; neither the missing values were removed from the dataset, nor were they replaced using certain values, that is, mean and median. Using missing values in the dataset can sometimes predict inaccurate results. Another drawback is that no optimization technique was used by the authors for the comparison of results.

### 3.8. Deepti Sisodia's Method

The authors have designed a machine learning model which can maximize the accuracy of the likelihood of diabetes in Indian patients. Three machine learning algorithms, namely, decision tree, that is, J48 [46], support vector machine [46], and naïve Bayes [47], are used for the classification of diabetes. Machine learning algorithms are run on the Pima Indians Diabetes Dataset, which is downloaded from the UCI repository. The authors have made use of Weka [48] to analyse the machine learning algorithms on PIDD. The main aim of using Weka by the authors is that, according to the given requirements, the tool can also be personalized. A 10-fold cross-validation technique is used for performing the experiments. Classifiers are run on the dataset after being undergone for 10-fold cross validation, and the evaluation parameters taken by the authors are precision, recall, accuracy, f-measure, and ROC curve. To check for the usefulness of the test, receiver operating characteristics are used by the author. The highest accuracy, that is, 76.3%, was achieved by the authors through a naïve Bayes classifier. Since there were no preprocessing techniques applied to the dataset, this method took very less time to execute, and experiments were conducted using Weka, which is also a very user-friendly tool.

### 3.9. M Orabi's Method

In this paper, the authors have made use of regression prediction to predict whether or not a person could be a candidate for having diabetes and at what age. To randomize the task of testing [49] and training, a rotation mechanism has been used by the author. The average of each iteration is calculated for comparison purposes. The dataset used by the authors was from the Egyptian National Research Centre. A questionnaire was prepared, which consisted of several questions for prediction purposes, and then the data was extracted using the SPSS tool and then imported into Excel sheets. The dataset contains 23 features which are age, gender, education, diabetic family member, smoker, cigarette number, exercising status, frequent exercise per week, exercise type, food type, healthy food status, number of basic meals, snacks status, snacks number, snacks type, regime status, blood pressure status, blood fat status, foot complications, neurocomplications, low vision status, and wound recovery status. The authors have preprocessed the dataset by cleaning, data reduction, and normalization of the dataset.

(1) Data cleaning consisted of the following steps:
  (i) Removing those rows from the dataset where the age of the people is less than 19 years and they are affected with type 1 diabetes.
  (ii) Removing those rows where null values are present as taking those values into consideration will affect consistency and accuracy.
  (iii) Removing the discrepancies by eliminating redundant rows from the dataset.
(2) Data integration [22] consisted of converting the data from the Egyptian National Research Centre by making use of the SPSS tool and then importing data into an Excel sheet. Since the authors have collected the data from a single source, there is no need for integration.
(3) Data reduction [25] consisted of eliminating those features from the dataset which are not required for prediction purposes. Only those features were taken into consideration by the author, which assisted them in early prediction.
(4) Data normalization shown in (7) requires the representation of the data into smaller values which was done by using min–max normalization equation by the author:
  (7) $$\begin{array}{c} \frac{\left(V_{i}-\text{min }A\right)}{\left(\text{max }A-\text{min }A\right)}, \end{array}$$
where *V*_*i*_ is the feature's current value, minA is the minimum value in the column, and maxA is the feature's maximum value.
(5) Data discretization converts the categorical value to a numerical value by assigning some weights to the value.

After the preprocessing [17] step, the dataset consisted of 9 significant features which were required for early prediction purposes, and then a decision tree classifier was applied to the dataset along with a customized rotation mechanism to make sure that every part is used for training as well as testing purpose. The method used by the authors is too slow as it takes a lot of time in data preprocessing, and the authors have made use of only one classifier, so there is no base for comparison with other machine learning algorithms.

### 3.10. O.M. Alade's Method

In this paper, the authors have worked on the Pima Indians Diabetes Dataset and made use of an artificial neural network [21] on the dataset for predicting diabetes. The authors have designed a neural network using the Bayesian algorithm and backpropagation method, and the neural network consists of four layers. To avoid any overfitting in the dataset, they made use of the Bayesian regulation algorithm [50], and for training purposes, the backpropagation [51] method was used. 70% of the dataset is used for training purposes, 15% for testing, and the remaining 15% for validation. Dataset is trained using MATLAB software, and the data is trained until a single and accurate output is displayed using regression graphs. The dataset contains 8 attributes; these 8 attributes form the 8 neurons of the input layer. Eight input neurons are the number of times a woman is pregnant, body mass index, diabetes pedigree function [9], age, plasma glucose concentration, blood pressure, insulin, and skin thickness. Then, two hidden layers with ten neurons are used. A hidden layer is a layer that receives input from the input layer and forwards output to the output layer. The output layer represents the results, and there is only one neuron present in the output layer. If the neuron in the output layer has a value equal to or greater than 0.5, the person is suffering from diabetes mellitus, otherwise not. After making use of the neural network to predict diabetes, a web-based graphical user interface was developed by the authors using JavaScript and NodeJS, where a user can enter their basic details and get to know whether they are suffering from disease or not.

## 4. Comparative Analysis

The task of predicting diabetes with utmost accuracy is still a very challenging task. There are so many features that contribute towards the prediction of diabetes, but it is a way difficult to identify those features and make use of those features to detect diabetes at an early stage. Thus, studying the characteristics and features for prediction purposes is a tedious process. Research has been undergoing for the last few decades, and the problem is still an open task. After studying the work done by various contributors and researchers, it has been concluded that we cannot predict which attributes from the dataset play an important role, and optimal feature selection cannot guarantee 100% accuracy. Classification methods used by most of the researchers are naïve Bayes, support vector machine, decision trees, random forest, k-nearest neighbour, multilayer perceptron, and logistic regression. Few researchers have made use of the recurrent neural network or deep learning and have devised a method that can correctly predict the instances.

In the year 2020, Kamrul Hasan et al. [36] proposed a methodology that consisted of feature selection, data preprocessing technique, and hyperparameter optimization using python. The authors made use of six classification algorithms, that is, random forest, k-nearest neighbour, decision trees, multilayer perceptron, AdaBoost [52], and extreme gradient boost [15]. The method proposed by the authors is a very tedious and lengthy process as the authors are calculating entropy at every step for decision tree and random forest and the main focus of the authors is on increasing AUC (area under the ROC curve), which came approximately near to 95% by using ensembling of AdaBoost and gradient boost.

In 2018, Zou et al. [27] devised a method in which the authors have worked on two datasets: one was publicly available Pima Indians Diabetes Dataset, and the other dataset was taken from a local hospital, that is, Luzhou in China, which consisted of approximately 68994 values. The authors have made of principal component analysis [23] and minimum redundancy maximum relevance features to make use of optimal feature selection and only a single feature; that is, blood glucose was also used for classification purposes. The method is very slow, and since the dataset was created by the authors themselves, we cannot predict how correct the evaluation parameters are predicted.

In 2017, Maniruzzaman et al. [53] presented a method that consisted of comparing linear, radial basis, and polynomial kernel for a Gaussian-based classification process using Laplace approximation. The authors have proposed a method in such a way that it can be used to classify linear and nonlinear data also. The main flaw of the model is the selection of the kernel for medical data representation in a correct manner. The method does not use any optimal feature selection methods, and it does not rank the features.

In 2019, Maniruzzaman et al. [37] devised a method in which he made use of logistic regression, probability value, and odds ratio to select the relevant features from the dataset. Dataset used by the authors was NHANES [54] (National Health and Nutrition Examination Survey) dataset which is the publicly available dataset. In this method, the authors have dropped the missing values, thus reducing the 9858 values to 6561 values. The process is very tedious since the authors are calculating probability value and odds ratio for feature selection.

In 2020, Jackins et al. [55] proposed a method in which the missing values were replaced by null values, and the authors calculated the amount of correlation between the features. If the two features have a high amount of correlation between them, one of the features can be dropped, and the other can be used for classification purposes. A correlogram matrix has been created, but the authors after calculation of correlation amongst attributes. The processing time of the method is very high.

In 2018, Sneha and Gangil [56] also calculated correlation amongst attributes, and the classification was done using the rapid miner tool. This method does not consider any other feature selection method [57], so it is difficult to analyse the accuracy as only the correlation calculation method is used by the author. In addition to this, the authors have not mentioned the public domain of the dataset. No filters were applied to the dataset, and we cannot predict diabetes accurately as the dataset may contain some missing values.

In 2019, Mohapatra et al. [58] proposed a method for the detection of diabetes using multilayer perceptron. The authors have split the dataset into training and testing. 550 values were used for training, the rest 218 were used for testing purposes, and the classification [59] has been done using the RStudio [14] tool. The disadvantage of the method is that no filters were applied to the dataset, nor any optimal feature selection method [60]. This method cannot be used for prediction purposes effectively.

In 2018, Sisodia and Sisodia [7] proposed a method in which a few machine learning algorithms, that is, naïve Bayes, support vector machine, and decision tree, were applied to the Pima Indians Diabetes Dataset [61]. The drawback of the method is that it is a very plain method used for classification purposes without any of the preprocessing methods applied to the dataset.

In 2016, Orabi et al. [62] proposed a method in which he used the dataset from the Egyptian National Research Centre. The authors have applied preprocessing technique to the dataset, thus reducing the dataset from 23 columns to 9 columns, and then the decision tree classifier with rotation mechanism was applied to the dataset. The method is too tedious since the authors have collected the dataset, then made use of the SPSS tool, and then imported it to an Excel sheet.

In 2018, Alade et al. [63] proposed a web-based graphical interface created using JavaScript and NodeJS [65], which asked the basic details of the user and predicted whether the person is suffering from diabetes or not. The authors made use of a neural network that outputs the results. In this method, the authors have only made assumptions based on certain parameters such as insulin and plasma glucose concentration. If the neuron outputs result less than 0.5, the person is not suffering from diabetes, otherwise yes. The main disadvantage of the method is that the authors have not taken any evaluation parameter to evaluate the results; only assumptions are made.

Every proposed method has its own set of drawbacks and advantages. All the methods are compared, and the comparison is shown in Table 1. The comparative analysis suggests that the best method so far is by the Kamrul Hasan et al.'s [36] method as it uses preprocessing techniques, feature selection methods, and hyperparameters tuning also, and the classification is being done by ensembling of AdaBoost and gradient boost algorithm. Other methods are not much efficient because they are also making optimal feature selection method, but a few of the methods lack preprocessing techniques, some of them are dropping missing values, and some of them are not using feature selection methods.

## 5. Discussions and Future Directions

All the methods proposed so far for the prediction of diabetes are focusing more towards feature selection strategy and few machine learning methods such as random forest, naïve Bayes, support vector machine, and decision trees, whereas only a few features are to be selected for prediction purpose. While studying all of these articles, the challenges that we faced are as follows:

1. The major challenge in prediction purpose was the absence of a larger dataset since the publicly available dataset contains only nine attributes, one being the class attribute. Time and effort are being spent on those features that have no potential to be selected for prediction purposes.
2. Most of the authors have dropped missing values from the standard dataset, which can affect the results as the size of the dataset decreases.
3. General machine learning algorithms are applied to the dataset; only one author has made use of AdaBoost and gradient boost technique. None of the authors has made use of the recurrent neural network or deep learning technology, which can help in increasing the efficiency. So, a method needs to be developed which can deliver more accurate results, has to be fast in terms of processing, and is more effective for the prediction purpose.

## 6. Recommendations

After conducting a survey of various articles on diabetic prediction models, we strongly recommend our study because of the following reasons:

- We have included recent articles.
- We have presented a comparative statement of major diabetic prediction models which will help other researchers to understand and evaluate the models.
- Advantages and disadvantages have been presented in Section 4.
- Various Strategies to predict diabetes have been discussed in the paper.

## 7. Conclusion

Based upon the comparative analysis and the above discussion, it can be concluded that Kamrul Hasan et al.'s [36] method is by far the best approach for diabetes prediction, as it is ranking features, selecting predominant features, filling missing values by median, and then tuning the hyperparameters as well. All the experiments were conducted using python. Although the accuracy achieved is only 78.9% by ensembling of AdaBoost and gradient boost, the AUC achieved is approximately 95%. A comparison of the three-feature selection technique and six machine learning classifiers has been made, and the ensembling of AdaBoost and gradient boost gave the best results.

## Figures and Tables

**Table 1:** Comparative analysis of diabetes prediction using machine learning methods.

S. no.	Method name	Number of datasets used	Name of the dataset	Data size	Speed	Does it rank features	CV protocol used	Evaluation parameters taken	Classifier used	Feature selection method	Number of features used	Classification accuracy	Year in which paper was published	Temporal interval
1	Kamrul Hasan	1	PIDD	768	Slow	Yes	5	Sn, Sp, and AUC	KNN, DT, RF, MLP, AB, XB, and NB	PCA, ICA, and CRB	6	78.9%	April 2020	2020-2021
2	Quan Zou	2	Luzhou and PIDD	68994, 768	Slow	Yes	5	Sn, Sp, ACC, and MCC	J48, RF, and NN	PCA and mrMR	11, 7	80.84%	November 2018	2018-2019
3	Nishith Kumar	1	PIDD	768	Fast	No	5 and 10	Sn, Sp, ACC, PPV, and NPV	GPC, LDA, QDA, and NB	Kernels	All	81.97%	December 2017	2016-2017
4	Maniruzzuman	1	NHANES	9858	Slow	No	2, 5, and 10	Sn, ACC, PPV, NPV, FM, and AUC	NB, DT, RF, and AB	LR	All	92.75%	January 2020	2020-2021
5	V. Jackins	1	PIDD	768	Fast	Yes	None	ACC	NB and RF	CRB	4	74.46%	November 2020	2020-2021
6	N. Sneha	1	PIDD	2500	Slow	Yes	None	Sn, Sp, ACC, PPV, NPV, PLR, NLR, and DP	SVM, RF, NB, DT, and KNN	CRB	11	82.3%	February 2019	2018-2019
7	S. Mohapatra	1	PIDD	768	Fast	No	None	ACC, TP, and TN	MLP	None	All	77.5%	September 2019	2018-2019
8	D. Sisodia	1	PIDD	768	Fast	No	None	Recall, precision, and ACC	NB, SVM, and DT	None	All	76.3%	December 2018	2018-2019
9	Orabi	1	Egyptian National Research Centre	Not mentioned	Slow	No	None	ACC	DT	Not mentioned	9	84%	2016	2016-2017
10	O. M. Alade	1	PIDD	768	Fast	No	None	ACC	NN	None	All	Only prediction was done	December 2017	2016-2017

## Data Availability

The data are available at https://www.kaggle.com/uciml/pima-indians-diabetes-database.

## Abbreviations:

PIDD: PIMA Indians Diabetes Dataset
Sn: Sensitivity
Sp: Specificity
AUC: Area under the curve
MCC: Matthews correlation coefficient
PPV: Positive predictive value
NPV: Negative predictive value
FM: F-measure
PLR: Positive likelihood rate
NLR: Negative likelihood rate
DP: Disease prevalence
TP: True positive
TN: True negative
KNN: K-nearest neighbour
DT: Decision tree
RF: Random forest
MLP: Multilayer perceptron
AB: AdaBoost
XB: Gradient boost
NB: Naïve Bayes
NN: Neural network
GPC: Gaussian process classification
LDA: Linear discriminant analysis
QDA: Quadratic discriminant analysis
PCA: Principal component analysis
ICA: Independent component analysis
CRB: Correlation-based
mrMR: Minimum redundancy maximum relevance
LR: Logistic regression.
